The article "Drug Packaging Management Based on the Effect of Medical Images on the Intracellular Polysaccharide Synthesis and Antivertigo Activity of Phalaenopsis" was published in 2021. Journal: J Healthc Eng.

# Drug Packaging Management Based on the Effect of Medical Images on the Intracellular Polysaccharide Synthesis and Antivertigo Activity of Phalaenopsis

**DOI:** 10.1155/2021/3793610

**Published:** 2021-08-04

**Authors:** Qiang Zhang, Li Zhang, Yue Li, Ming Ye

**Affiliations:** ^1^School of Biological Sciences and Engineering, North Minzu University, Yinchuan 750021, Ningxia, China; ^2^School of Food and Biological Engineering, Hefei University of Technology, Hefei 230009, Anhui, China; ^3^The Administration Department of Nosocomial Infection of the First Hospital of Lanzhou University, Lanzhou, Gansu 730000, China; ^4^Hangzhou Huatai Testing Technology Co. Ltd.,, Hangzhou 310000, Zhejiang, China

## Abstract

Many clinically important drugs come directly or indirectly from higher plants. People are increasingly aware of the role of the human immune system in maintaining good health. Diseases related to physical dysfunction, such as vertigo, have attracted increasing attention from medical researchers and clinicians. In this paper, some compounds isolated and identified from medicinal fomes showed promising antivertigo properties. Medical images were used to classify and synthesize polysaccharides in the management of drug subpackages of *Cladosporium* intracellular polysaccharides. The scientific explanation of how these compounds work in animal and human systems is increasing exponentially. Studies have found that all of these compounds can enhance the innate and adaptive immune responses of the host and activate various immune cells that are important for maintaining homeostasis, such as host cells and chemical messengers, triggering complement and acute phase reactions. The antivertigo compounds derived from the intracellular polysaccharides of Phellinus mucronatus had an activity interference of 35% without drug subpackage. Although the antivertigo activity of many intracellular polysaccharides from Fovea xylostella can reach 86%, only a few of them have been proved to have antivertigo activity. In addition, they can be considered as multicytokine inducers that can induce the expression of various immune-regulatory cytokines and cytokine receptor genes. Lymphocytes that control antibody production and cell-mediated cytotoxicity are also stimulated.

## 1. Introduction

In recent years, it has been found that the intracellular polysaccharides of fomes trochoidum can improve the function of immune cells and immune organs. Therefore, it has a certain regulatory effect on in vivo and in vitro immunity. In this paper, the effect of blockchain technology on the synthesis of polysaccharides and antivertigo activity of microorganisms was studied. At present, many scholars use the intracellular polysaccharides of *Cladosporium* to synthesize effective biological applications in the future.

The article "Drug Packaging Management Based on the Effect of Medical Images on the Intracellular Polysaccharide Synthesis and Antivertigo Activity of Phalaenopsis" was published in 2021. Journal: J Healthc Eng.

Research at home and abroad has made great achievements in different branches, such as Wang. Through research, it was found that the intracellular polysaccharide of fomes xylatum can act on spleen lymphocytes of mice in a certain range, to improve its antivertigo activity [1]. Moreover, the spleen lymphocyte proliferation index and other evaluation indexes showed that the synthesis of intracellular polysaccharides and antivertigo activity of the molecularly modified polysaccharides were higher than those of the molecularly modified polysaccharides, and the sulfated polysaccharides were more effective than the polysaccharide modified polysaccharides stronger [2]. Zheng found that the purified intracellular polysaccharide could prevent the recognition and adsorption of enveloped viruses such as HSV-1, HSV-2, and influenza A virus in cells, playing a strong antiviral role [3]. Li proposed that the intracellular polysaccharide of *Cladosporium* could not block the penetration of the virus that had been bound to the host cell, but at the initial stage of the virus's effect on the host cell, the binding process between the virus and the cell could be blocked by the intracellular polysaccharide of *Cladosporium*, thus reducing the probability of cell infection [4]. Yao thought that the intracellular polysaccharide of the fungus had no antithrombin activity, so it would not have side effects on the cells. Therefore, the intracellular polysaccharide of *Cladosporium* xylatum can be used as an effective antiviral drug in the future [5,6].

Ho sprayed sodium sulfite on the leaves of *P. xylostella* according to the different growth stages and different dosages. It was found that the sugar content increased the most in the fruit expansion stage, and the soluble sugar content also increased significantly. Too high sodium sulfite concentration would lead to the decrease of polysaccharide content [7,8]. Feng used the encapsulation image experiment to change the sugar content in the environment with different concentrations of polysaccharide reagent to observe the sugar enrichment ability of *Porus xylostensis*. It was found that the sugar content and total sugar content of *Porus xylostensis* increased after sugar enrichment, indicating that the sugar content in the environment can effectively improve the sugar enrichment of *Porus xylostensis* [9,10]. Cui used GC to analyze the polysaccharide of rich sugar *Grifola frondosa*. The results showed that the ratio of mannose, glucose, and galactose was 3.3 : 2 and 3.3 : 1 [11]. Combined with the acidic and neutral polysaccharides, it was found that the content of uronic acid may affect the degree of sugar enrichment. In addition, Yang found that different methods of sugar enrichment may have a certain impact on the monosaccharide composition. The determination of monosaccharide composition is helpful to determine which functional groups in polysaccharides react with sugars and effectively determine which polysaccharides are more suitable for the preparation of polysaccharides [12]. The above studies focus on the effects of bacterial sugars on the bacteria themselves, and the findings are still experimental. Based on this, this paper uses blockchain drug packaging imaging technology to conduct a comparative study of the relationship between intracellular polysaccharide synthesis and antivertigo activity.

The article "Drug Packaging Management Based on the Effect of Medical Images on the Intracellular Polysaccharide Synthesis and Antivertigo Activity of Phalaenopsis" was published in 2021. Journal: J Healthc Eng.

In this paper, the effects of blockchain technology on the synthesis of intracellular polysaccharides and antivertigo activity of Porus unguiculatus were studied. In this paper, monosaccharide, monosaccharide, or monosaccharide was used to synthesize polysaccharides. This method almost did not change the spatial structure of polysaccharides and maintained most of the biological activities of polysaccharides. In this paper, the antivertigo activity of cells with manganese ions as the core was studied.

## 2. *Porus xylostensis* and Drug Packaging Image Technology

### 2.1. Synthesis of Intracellular Polysaccharides

As a new kind of bioactive polysaccharide, the intracellular polysaccharide of fomes xylostella has a certain antitumor activity in vitro. The extracellular polysaccharides produced by the protomycetes and cells of *Cladosporium* xylatum have an inhibitory effect on human hepatoma cell HepG2, and the caspase-3 enzyme activity is significantly increased in the process of action, which indicates that the intracellular polysaccharides of *Cladosporium* xylatum may achieve the purpose of inhibiting tumor cell activity by inducing mitochondrial apoptosis [13]. To explore the effect of salt stress on the antitumor activity of EPS, Lumiao chose HT-29 and LoVo, considering that EPS mainly plays a role in the human intestinal tract. The results showed that the extracellular polysaccharide of *P. xylostensis* under salt stress and normal culture conditions could effectively prevent the proliferation of tumor cells, and the effect of extracellular polysaccharide of *P. xylostensis* under salt stress was stronger than that of intracellular polysaccharide of *P. xylostensis* under normal culture conditions [14]. Both foliar spraying of high sugar and environmental high sugar could increase the sugar content in the plant but had a greater impact on the polysaccharide content in the mycelium, and the obtained polysaccharide content was less [15]. In addition, there are high requirements for sugar application conditions. In addition to considering the growth state and the dosage of polysaccharide reagent, we should also pay attention to the influence of plant health state, environmental pH, species, soil conditions, and environmental adsorption on the sugar transformation in *P. xylostella* [16].

The article "Drug Packaging Management Based on the Effect of Medical Images on the Intracellular Polysaccharide Synthesis and Antivertigo Activity of Phalaenopsis" was published in 2021. Journal: J Healthc Eng.

At present, the mechanism of stress resistance response and the mechanism of polysaccharide synthesis are still under further study [17]. A comprehensive understanding of the enzymes and genes related to the biosynthesis of intracellular polysaccharides of *P. xylostella* is helpful to construct high-yield *P. xylostella* species, to realize the large-scale production of intracellular polysaccharides of *P. xylostella*, to meet the growing demand of consumers for food and medical treatment. In recent years, a number of studies have shown that the intracellular polysaccharides of cladosporus cladosporus have antioxidant, antibacterial, and anti-inflammatory, antivirus, antitumor, and immunomodulatory functions [18]. Therefore, the intracellular polysaccharides of Cladosporus cladosporus are gradually developed and applied in food, medicine, and other fields, which has a good development prospect [19]. The research on blockchain in academic circles is becoming one of the focuses of attention of many disciplines/directions, such as software engineering, computer science, network and information security, industrial manufacturing, and mathematics [20].

For the pathway of polysaccharide synthesis, there have been some reports on the pathway of polysaccharide synthesis in bacteria, but few reports on fungal polysaccharides [21]. However, the basic pathway of polysaccharide synthesis of fungi and bacteria has a certain similarity, which is divided into precursor supply, synthesis initiation, monosaccharide polymerization, and polysaccharide output [22]. Some researchers used the isotope tracer methods to study the pathway of polysaccharide synthesis, and others used molecular means such as gene overexpression to carry out related research [23].

### 2.2. High-Efficiency Gel Permeation Chromatography Method for the Synthesis of Medical Image Polysaccharides

HPGPC (high-performance gel permeation chromatography) is a method for studying the molecular weight and distribution of polysaccharides. High-performance gel permeation chromatography (GPC) and size exclusion chromatography (GC) were used to separate the sugar polysaccharides to produce polysaccharides of different molecular weights. In this paper, *Artemisia sphaerocephala* polysaccharides were separated by size exclusion chromatography. It was found that the low molecular weight (1.026∼1.426) × 104 g/mol showed a rigid structure, and the high molecular weight (2.268∼4.363) × 104 g/mol showed a compact DNA structure, as shown in Figure 1.

The article "Drug Packaging Management Based on the Effect of Medical Images on the Intracellular Polysaccharide Synthesis and Antivertigo Activity of Phalaenopsis" was published in 2021. Journal: J Healthc Eng.

In addition, the molecular weight of tea polysaccharides was determined by high-performance gel permeation chromatography. It was found that polysaccharides with a low molecular weight of 1.3 *∗* 104 Da may exhibit higher antioxidant capacity [24]. The determination of the molecular weight of polysaccharides is helpful to analyze the relationship between the structure and activity of polysaccharides. However, the chemical synthesis method needs to prepare polysaccharides in an acidic environment, and the degradation of the polysaccharide chain in an acidic environment leads to the decrease of molecular weight, which affects the molecular weight distribution [25]. Therefore, the determination of the molecular weight of polysaccharides should be combined with other analytical methods. The acetylation of carboxylic acid sugar ether with *Ganoderma lucidum* polysaccharide can produce a polysaccharide with a c-sec structure, which can significantly increase the in vitro antitumor activity and improve the bioavailability. Compared with the transformation method of fomes, it is more simple and efficient. The sugar elements in the environment can be absorbed by *Porus xylostensis*, form glycogen anion or monosaccharides (SE0) through oxidation and reduction in vivo, and combine with polysaccharides in the cell wall or transport into cells through the cell membrane for enrichment [26]. In recent years, there are increasing researches on adding polysaccharide reagents to the culture medium for fungi and bacteria [27].

### 2.3. Blockchain Technology and Encryption Algorithm

Due to the openness and transparency of blockchain, synthetic data and network node addresses are facing serious privacy leakage problems. In terms of performance, the performance of existing blockchain platforms is far lower than that of traditional centralized systems, which is difficult to be applied in large-scale synthetic scenarios; in terms of interoperability, a large number of blockchain applications based on different underlying technologies cannot conduct trusted data flow and value exchange [28]. In recent years, ICSE, CCS, podc, DSN, and other well-known conferences have included the topic of blockchain, and international conferences with blockchain as the theme, such as IEEE Blockchain and BlockSys, have also begun to appear in large numbers. It can be seen that this field is showing the research heat of accelerating temperature rise. With the in-depth development and wide application of blockchain, it also faces increasingly technical challenges.

The article "Drug Packaging Management Based on the Effect of Medical Images on the Intracellular Polysaccharide Synthesis and Antivertigo Activity of Phalaenopsis" was published in 2021. Journal: J Healthc Eng.

Through the tree structure to create multiple subchains, a large number of computing processes are transferred to the subchains to reduce the synthesis load of the Ethereum main chain, to improve the performance of the blockchain. However, plasma needs nodes to constantly verify the subchain to ensure the security of assets, and when malicious nodes refuse to provide synthetic data, they will face the unavailability of data, and large-scale exit of nodes may cause congestion in the main chain. Similarly, rollup (divided into ZK rollups and optimal rollups) manages the data transmission between the subchain and the main chain through the smart contract packages and encrypts a large number of synthetic state changes and provides data availability proof for the main chain without submitting all synthetic data. ZK snarks are used to verify new blocks to avoid the challenge period set for detecting malicious composition in plasma. However, generating a ZK snark on a block-by-block basis requires a high computational cost. The optimal rollup should provide an error proof for the verifier to validate the published blocks within a 1-2 week challenge period. If the block turns out to be invalid, it will be rolled back. If there are no nodes to send error proofs, there is no need to validate the block. However, this will lead to no synthesis confirmation before the end of the challenge period, and it is difficult to ensure the safety of synthesis. At present, both schemes are still in the early stage of research and development and need to overcome the challenges of security and the length of final confirmation of synthesis in blocks. Encapsulation channel is to establish a channel between different users or between users and services, move a large number of calculations out of the chain, and store the final results on the blockchain after the calculation is completed and confirmed by multiparty signature. Packaging channels can be simply divided into unidirectional packaging channels and bidirectional packaging channels according to the synthesis mode. The unidirectional encapsulation channel only supports unidirectional encapsulation and cannot support synthetic bidirectional transmission, so its application is very limited. The existing packaging channel schemes are mainly two-way channels, and the typical applications include a lightning network.

#### 2.3.1. Basic Application Algorithm of Blockchain

Lightning network is an encapsulation system built for the defects of low throughput and difficulty to support small amount synthesis of the bitcoin blockchain, which enables users to synthesize in a low-cost and high-throughput environment. Users only need to record the synthesis results of the encapsulated channels on the blockchain regularly and do not need to submit all synthesis results, to improve the throughput of the bitcoin blockchain:

(1) $$\begin{array}{c} \text{HINE}=\sum_{i,j}^{N}f\left(X_{ij}\right){\left(v_{i}^{T}v_{j}+b_{i}+{\text{KL}}_{j}-\log\left(X_{ij}\right)\right)}^{2}. \end{array}$$

If one node fails in the synthesis process, the whole channel will be interrupted, and the lightning network will face the problem of single-point failure. In addition, the synthesized polysaccharides are limited by the locking number of nodes, which makes it difficult for the lightning network to support large-scale synthesis. In the latest research progress, the lightning network has tested the multipath encapsulation scheme, which divides the large sum synthesis into several small sum syntheses and arrives at the synthesis party through different routes:

(2) $$\begin{array}{c} \sigma_{ikjl}=\left\{\begin{array}{cc} \frac{n}{\Delta_{ikjl}}\sqrt{\sum_{s=1}^{n}{\left(x_{ik}\left(\varepsilon \right)-x_{jl}\left(\varepsilon \right)\right)}^{2}\Delta_{ikjl}\left(\varepsilon \right)}, & \Delta_{ikjl}>0,\\ 0, & \Delta_{ikjl}<0. \end{array}\right. \end{array}$$

*σ* represents a composite relationship between target nodes and targets, where *ε* represents the composition operator between relations, *X* represents the node type, and Δ represents the relationship type. In this way, the packaging problem of large amount synthesis can be solved. Most bidirectional encapsulation channel schemes need to establish a channel for both sides of the synthesis, and the establishment of the channel needs to rely on an intermediate node, which is contrary to the concept of blockchain decentralization. For this reason, Perun introduces a virtual encapsulation channel technology to directly establish a virtual channel for both sides of the synthesis without introducing intermediate nodes:

(3) $$\begin{array}{c} {\text{Perun}}_{ij}=\frac{e^{b_{ij}}}{\sum_{k}e^{b_{ik}}},\\ u_{\left(j|i\right)}=w_{ij}A_{i}. \end{array}$$

*A* represents all possible situations in the channel. In the encapsulation channel scheme, the images of both sides need to be locked for a period of time. When malicious nodes continue to initiate synthesis, it may cause images on a path (multiple encapsulation channels connected) to be locked, thus causing sad attacks. In view of this, a new measurement method is proposed for images locked in the channel to solve the problem of too long image locking time and resist the possible sadness attack:

(4) $$\begin{array}{c} W_{t}=\tan h\left(w_{c}x_{t}+u_{c}\left(r_{t}\Theta h_{\left(t-1\right)}\right)+b_{c}\right),\\ Q_{t}=z_{t}\Theta h_{t-1}+\left(1-z_{t}\right)\Theta h_{t}, \end{array}$$

where *Q, I*, and *w* denote the area of measurement. After the introduction of the image warehouse, two steps are added between the peer and deployment node to push and pull the image to the warehouse:

(5) $$\begin{array}{c} R_{\text{ssim}}=A-\frac{\left(2\mu_{x}\mu_{y}+C_{1}\right)\left(2\sigma_{xy}+C_{2}\right)}{\left(\mu_{x}^{2}+\mu_{y}^{2}+C_{1}\right)\left(\sigma_{x}^{2}+\sigma_{y}^{2}+C_{2}\right)},\\ E_{1}^{ij}=\cos\left(S_{1}^{i},S_{2}^{j}\right). \end{array}$$

Native peer initiates the task of image compilation and container creation to the Docker daemon through the Docker SDK. Now, chain code instantiation is divided into two processes: image compilation and container creation. Image compilation is still completed through the peer, but the image is pushed to the image warehouse in the cluster; to create a container, you need to integrate Kubernetes SDK in the peer to complete the deployment of the container. The work node that obtains the deployment task pulls the chain code image from the remote warehouse and creates the chain code instance. According to the similarity between blockchain and function computing, service chain code is the most potential component of the fabric based on function computing. Failure of some chain code containers does not affect the entire blockchain network. Make fabric if you need to calculate a new configuration. Pull up the container again. This capability of the fabric makes it possible to realize the computational management of the chain code container function. Fabric chain code is a component that only provides computing services. All its data comes from peer service, which meets the requirement of stateless code for function computing service. To complete the chain code calling task, we need to go through the process of chain code installation and instantiation in turn. After instantiation, the chain code container of the peer server is always in a running state waiting to be called. Only when the chain code is upgraded or an internal error occurs in the chain code itself does the chain code container end:

(6) $$\begin{array}{c} \Delta_{ikjl}=\sum_{\delta =1}^{n}\Delta_{ikjl}\left(\varepsilon \right),\\ \log_{m}n\leq \text{depth}\leq \log_{\left\lceil m/2\right\rceil }\left(\frac{n}{2}\right)+1. \end{array}$$

The article "Drug Packaging Management Based on the Effect of Medical Images on the Intracellular Polysaccharide Synthesis and Antivertigo Activity of Phalaenopsis" was published in 2021. Journal: J Healthc Eng.

#### 2.3.2. Function Computing Service Management Chain Code

The first thing to do is to change the life cycle of the chain code. The chain code container is required to instantiate and start again when it is called, and exit when it is called. Whether a functional computing service or blockchain service, deploying user code needs to solve the code compilation problem. The compilation of fabric chain code is a complex process, which can not prepare the code in advance and upload the dependency package directly as the function computing service. At present, the industry or community function computing service can not complete the compilation of fabric chain code:

(7) $$\begin{array}{c} \text{Docker}=\frac{\text{TP}+\text{TN}}{\text{TP}+\text{TN}+\text{FP}+\text{FN}},\\ \text{Kubernetes}=\frac{\text{TP}}{\text{TP}+\text{FP}},\\ \text{Knative}=\frac{\text{TP}}{\text{TP}+\text{FN}}. \end{array}$$

In view of the actual situation, this paper uses the method of simulating function computing service to carry out the experiment. The user code deployment of a function computing service can be divided into image compilation, distribution, deployment, and other processes. Taking the native function computing service as an example, the user code is compiled into a Docker image and stored in the remote image warehouse. The event triggers the computing node to pull the image from the warehouse, start the instance, and exit after completing the task. Fabric peer has the ability of encoding and decoding the chain code images. The Kubernetes deployment scheme designed in this paper also completes the distribution of chain code images in the cluster, so only the scheduling task of the chain code instances needs to be modified. By adding the serverless field in the CDs structure and adding the serverless tool global parameter under the chain code install subcommand, the running mode of the chain code container can be changed and the scheduling task can be completed. The chain code with the serverless parameter is started as follows:

(8) $$\begin{array}{c} v_{t1}=\left(w_{1}^{1},w_{2}^{1},w_{3}^{1},w_{4}^{1},w_{5}^{1}\right),\\ N\geq n+\frac{n}{2}+\frac{n}{4}+\cdots +1=2n-1, \end{array}$$

where *W* is the path and *V* is the edge. Introducing a serverless multitenant network shared computing pool can significantly reduce the deployment and operation costs of the blockchain and reduce the cost threshold of users in the chain [29]. At the same time, the computing resource pool is transparent to users, sharing resources and ensuring data security privacy, which has the same meaning as above:

(9) $$\begin{array}{c} \left\{\begin{array}{c} \sigma =\prod_{i=s_{1}}^{s_{l}}\sigma_{i}^{v_{i}}=\prod_{i=s_{1}}^{s_{l}}H{\left(v\left\|i\right.\right)}^{v_{i}}u^{v_{i}s_{i}},\\ \mu =\sum_{i=s_{1}}^{s_{l}}v_{i}f_{i}, \end{array}\right.\\ 2{\left\lceil \frac{m}{2}\right\rceil }^{d-2}\times \left\lceil \frac{m}{2}\right\rceil \leq n\leq m^{d-1}\times m. \end{array}$$

The fabric blockchain platform is a complex distributed system with the high complexity of cloud deployment:

(10) $$\begin{array}{c} {\text{fabric }}_{i}={\left(H\left(f_{i}\right)\cdot u^{f_{i}}\right)}^{x}|\sigma_{i}\in G,i=1,2,\ldots ,n,\\ e\left(\sigma ,g\right)\overset{N}{=}e\left(\prod_{i=s_{1}}^{s_{l}}H{\left(v\left\|i\right.\right)}^{v_{i}}\cdot u^{\mu },v\right). \end{array}$$

In this paper, fabric components are divided into static and dynamic. Static components such as ca, orderer, and peer constitute the main basic framework of distributed systems. The static components can be started when the fabric network is deployed (excluding the nodes dynamically added in the running).

The article "Drug Packaging Management Based on the Effect of Medical Images on the Intracellular Polysaccharide Synthesis and Antivertigo Activity of Phalaenopsis" was published in 2021. Journal: J Healthc Eng.

## 3. Experiment

### 3.1. Content

In this paper, the effect of medical imaging technology on the synthesis of intracellular polysaccharides and antivertigo activity of *S. holier* was studied. This article summarizes 36 applications of medical imaging technology in the field of microbial and bacterial research in the past five years. It is found that the synthesis and antivertigo activity of intracellular polysaccharides are mainly affected by intracellular manganese ions. Therefore, this article mainly studies the effect of manganese ions on the antivertigo activity of cells.

### 3.2. Process

This experiment is mainly composed of polysaccharide synthesis, sorting, conveyor belt, and drug rack. *Porus xylostensis* for polysaccharide synthesis is installed between the cell membrane, which is responsible for transporting the drugs into the intercellular space and placing them on the drug rack. Or according to the drug list requirements provided by the upper computer system, the drugs are identified by the camera, and the drug coordinates are obtained, and then the specified drugs on the cell membrane are transported to the intercellular space; each drug collection site has a sorter that receives data from the computer at the top to retrieve drug list numbers, drug numbers, quantities, and more. If there is a drug to pass through, first identify the type and then transport the drug. This system ensures the accuracy of drug delivery through secondary identification and transport of drugs by prescription synthesis and classification. The polysaccharide was prepared by using glycosylate, oxychlorinated sugar, and organic polysaccharide complex as polysaccharide reagent.

Using monosaccharides, monosaccharides, or monosaccharides as a polysaccharide reagent to synthesize polysaccharides, this method almost does not change the spatial structure of polysaccharides and maintains most of the biological activities of polysaccharides. Taking the reaction of the polysaccharide system of HNO_3_ and BaCl_2_ as an example, BaCl_2_ has strong coordination with hydroxyl, enhances the nucleophilicity of oxygen, and the sugar element binds to the hydroxyl of polysaccharide to form a stable single complex. There are differences between the Kubernetes environment and ordinary Docker environment in image management and running environment. This section evaluates the performance of the modified chain code called by the speed of the task completion time under the same amount of tasks. The test benchmark is the chain code completion time based on the Docker running environment. The test environment is a dual organization single node deployment environment, and the solo algorithm is adopted. The chain code call is encapsulated by script, the call times are specified by parameters, and the start and end times of the call are output. In Docker and Kubernetes environments, the performance of chain code deployed by Kubernetes is similar to that of Docker chain code. In addition, the number of successful calls of Docker and Kubernetes chain codes under 100 calls is set to 18.4 and 19, respectively, so that the success rate of the two calls is similar.

The article "Drug Packaging Management Based on the Effect of Medical Images on the Intracellular Polysaccharide Synthesis and Antivertigo Activity of Phalaenopsis" was published in 2021. Journal: J Healthc Eng.

The core of the design of a machine vision-based drug extraction system is to identify and locate drugs. In this paper, a drug identification algorithm based on the fusion of local features and the mean shift algorithm is proposed. First of all, the polysaccharide synthesis of fomes xylostella identified and matched the drugs on the cell membrane through the AKAZE algorithm and then transported them to the conveyor belt; sorting fomes xylostella identified the dynamic drugs on the conveyor belt through the improved mean shift algorithm and then transported them to the drug-taking place to complete the drug-taking function of the whole system. To overcome the influence of environmental factors such as light intensity and ensure the accuracy and real-time performance of the mobile terminal in the process of drug identification, the AKEZE algorithm is used to identify and match the drugs. After obtaining the location of drugs, further trajectory planning is carried out to complete the transportation and placement.

## 4. Experimental Results and Discussion

In this section, we first analyzed the advantages of blockchain in drug packaging images and then simulated the relationship between the content of intracellular polysaccharides and antivertigo activity by manganese ion concentration.

### 4.1. Blockchain Protocol for the Drug Packaging Image

Blockchain technology and ROMA (application and data integration platform) integration platform are integrated to jointly solve the challenges of drug packaging image. Through the above research and practice, we can see that blockchain technology can be applied to drug packaging image and application framework, but the specific application is not discussed in detail, and whether blockchain and existing mature technology will be more suitable for drug packaging image is not discussed. Rama integration platform has not been analyzed and summarized by the academics and then sublimated to the theoretical level to supplement the existing theory and better guide future practice.

The article "Drug Packaging Management Based on the Effect of Medical Images on the Intracellular Polysaccharide Synthesis and Antivertigo Activity of Phalaenopsis" was published in 2021. Journal: J Healthc Eng.

As shown in Figure 2, P2P propagation and ROMA are conducive to eliminating data islands and promoting data sharing. Point-to-point propagation realizes that all nodes share the data, and technology endorsement realizes the trust between nodes. Detrusting helps to promote the trust between each node and break the data island. Through the management of public cloud, private cloud, edge, and other nodes, ROMA console can get through the biological services, data devices, and data islands on and off the cloud and realize multicloud collaboration and cross-cloud and cross-regional interoperability; ROMA integration platform provides 30 + heterogeneous data sources and predocking with mainstream IT systems, MODBUS, opc-ua, and other common industrial protocols to promote data sharing. Cryptography algorithms, traceability, and distributed storage are conducive to the security of biological shared data.

### 4.2. Effect of Key Genes on Polysaccharide Synthesis of Fomes Xylostella

Firstly, on the basis of multiomics data and bioinformatics analysis, the target genes were screened by MATLAB analysis software and tools to obtain the key genes with research value; then, the function of the key genes was verified by silencing, heterologous expression, and other molecular biological methods. By constructing gene expression vectors with different functions, the gene level, protein level, and enzyme activity level were verified in the model strain; finally, through homologous expression in this species and in-depth analysis of the products, we can obtain a variety of results such as the amount of gene expression, products, components, and biological activity analysis and comprehensively analyze and verify from the product level, to obtain the key genes that promote the synthesis of polysaccharides. The continued development of gene cluster mining technology has greatly facilitated the study of new functional genes, the discovery of new natural products, and the analysis of biological functional information.

The article "Drug Packaging Management Based on the Effect of Medical Images on the Intracellular Polysaccharide Synthesis and Antivertigo Activity of Phalaenopsis" was published in 2021. Journal: J Healthc Eng.

As shown in Figure 3, the content of polysaccharides is different, which may be related to the purity, molecular weight, monosaccharide composition, and extraction process of polysaccharides. The microwave-assisted reaction time of polysaccharides and microwave-assisted reactions can be reduced. There are two reaction mechanisms for the use of chlorine oxidized sugar (seocl2) as a polysaccharide reagent. One may react with two cis-hydroxyl groups on the polysaccharide to form a monosaccharide ester compound to form a polysaccharide. Another method of polysaccharide synthesis: the content of polysaccharide (*μ* g/g) and the feed ratio of polysaccharide (sepap) PAP : H_2_SeO_3_ = 1 solid superacid was 49.37 mg and stirred at 78.39°C for 134.84 min.

As shown in Table 1, although there are many kinds of bacterial polysaccharides and their structures are complex and changeable, their biosynthesis mechanisms are similar. The key gene mining using the third-generation sequencing technology is a practical application model of bioinformatics analysis. After the multiomics analysis of the genome, transcriptome, and proteome, we use the program in the table and database to compare the genes and preliminarily determine the function of unknown genes in the organism, to provide direction for the discovery of target genes. A gene related to exopolysaccharide synthesis (epsN) was identified by bioinformatics analysis, which indicated that epsN played a key role in the pathway of exopolysaccharide synthesis, and was verified by molecular blockchain technology.

### 4.3. Effect of Manganese Ion on the Content of Polysaccharides in Fomes Xylostella

As shown in Figure 4, with the increase of manganese ion concentration, the intracellular polysaccharide content of fomes xylostensis increased at first and then decreased. When the mass concentration of manganese ion was 0.005 mg/L, the intracellular polysaccharide content of fomes xylostensis increased. When the environment is suitable, it is conducive to the production and storage of intracellular polysaccharides, so that they can be secreted under stress. When the manganese ion concentration was more than 0.005 mg/L, the content of intracellular polysaccharides decreased, which was caused by the cell rupture and the secretion of intracellular polysaccharides.

With the increase of manganese ion concentration, the content of intracellular polysaccharides increased first and then decreased. When the mass concentration of manganese ion was 0∼0.005 mg/L, it could promote the synthesis of intracellular polysaccharides, which was conducive to reserve a large amount of intracellular polysaccharides, so that once the cell growth was stressed, it could secrete a large amount of intracellular polysaccharide to protect the cell body. Bioinformatics analysis is to analyze and predict the functional segments of potential genes through the bioinformatics analysis website and software after sequencing the whole genome of the studied species and then focus on the target gene cluster. Since the process of polysaccharide synthesis is complex and involves many important enzymes and genes, we perform integrated analysis and prediction of polysaccharides before digging up some important genes for polysaccharide synthesis and experimenting. With the rapid development of big data, the constantly updated database provides us with sufficient convenience for data mining.

The article "Drug Packaging Management Based on the Effect of Medical Images on the Intracellular Polysaccharide Synthesis and Antivertigo Activity of Phalaenopsis" was published in 2021. Journal: J Healthc Eng.

As shown in Figure 5, with the increase of manganese ion concentration, the intracellular polysaccharide content of a single cell increased first and then decreased. The results of antivertigo activity showed that there was a significant difference in the content of intracellular polysaccharides among different manganese ion concentration groups (*F* = 138.836, *P* < 0.01). Duncan's multiple comparison results showed that the intracellular polysaccharide content of a single cell was significantly higher than that of other groups when the mass concentration of manganese ion was 0.005 mg/L, and there was no significant difference when the mass concentration of manganese ion was 0.5∼5 mg/L.

As shown in Table 2, with the increase of manganese ion concentration, the extracellular polysaccharide content of a single pore showed an increasing trend. When the mass concentration of manganese ion was 5 mg/L, the extracellular polysaccharide content of a single pore reached the peak value of 0.095 PG cell-1. The results of antivertigo activity showed that there was a significant difference in the content of exopolysaccharides among different groups (*F* = 330.255, *P* < 0.01). Duncan's multiple comparison results showed that there were significant differences among the groups. When the mass concentration of manganese ion was 5 mg/L, the extracellular polysaccharide content of a single cell was significantly higher than that of the other groups.

As shown in Figure 6, with the increase of manganese ion concentration, the carotenoid content of Cladosporus cladosporus increased first and then decreased. When the mass concentration of manganese ion was 0.005 mg/L, the promoting effect was the strongest, and the mass concentration of carotenoids was 0.19 mg/L. The results of antivertigo activity showed that the carotenoid content of different groups was significantly different (*F* = 150.695, *P* < 0.01). Duncan's multiple comparison results showed that there were significant differences among the groups. When the mass concentration of manganese ion was 0.005 mg/L, the difference was the most significant.

The article "Drug Packaging Management Based on the Effect of Medical Images on the Intracellular Polysaccharide Synthesis and Antivertigo Activity of Phalaenopsis" was published in 2021. Journal: J Healthc Eng.

As shown in Figure 7, the extracellular polysaccharide of fomes xylostensis showed an increasing trend with the increase of manganese ion concentration. When the manganese ion concentration was 0.005 mg/L, the synthesis amount of extracellular polysaccharide was 2.3 times that of the control group, and when the mass concentration of manganese ion is 5 mg/L, the content of extracellular polysaccharide is 3.36 times higher than that of the control group. Therefore, compared with the appropriate concentration, the stress environment formed by a high concentration of manganese ions can promote the secretion of exopolysaccharides to protect the cell body from injury. Therefore, we should pay attention to control the concentration of manganese ions in a reasonable range in directional cultivation.

As shown in Figure 8, under the stress of high concentration of polysaccharides, the allelopathic effect increased with the culture time, the thylakoid structure of the fungus was broken, the photosynthetic system of the algae was seriously damaged, the photosynthetic activity and photosynthetic efficiency were reduced, the synthesis of polysaccharide was inhibited, and the secretion and dissolution of polysaccharide were further promoted, resulting in a sharp decrease in the content of intracellular polysaccharide and a sharp increase in the content of soluble extracellular polysaccharide the phenomenon of the dramatic increase.

### 4.4. Discussion

In this paper, based on the existing research, according to the problems of drug packaging image, combined with the technical architecture of blockchain and ROMA integration platform, the overall architecture of drug packaging image system based on blockchain technology and ROMA integration platform is constructed, and how to embed and apply the two technologies to drug packaging image is mainly discussed, to bring new ideas for drug packaging image. Smart contracts and synthetic records help to clarify the power responsibility relationship among various departments. Based on the smart contract technology, the rights and responsibilities, the design system, and standard specifications are defined from the perspective of the structure and operation in the process of data sharing, and the contract level rule set is formed. Finally, the work technology flow is embedded into the system platform to help solve the problem of unclear rights and responsibilities between departments. In addition, each transaction is recorded on the block, such as data request, data provision, and data evaluation, which can be traced back to the synthetic record, effectively avoiding the problem of interdepartmental rights and responsibilities.

The article "Drug Packaging Management Based on the Effect of Medical Images on the Intracellular Polysaccharide Synthesis and Antivertigo Activity of Phalaenopsis" was published in 2021. Journal: J Healthc Eng.

For a long time, the performance of blockchain in terms of throughput, data storage, and scalability is far less than that of traditional databases. The performance problem has become a bottleneck that the blockchain must break through when it is widely used. For this reason, researchers have proposed a number of performance optimization schemes for block capacity, network communication, block time, and other performance factors. According to the implementation and analysis of existing performance optimization schemes, existing research work focuses on improving and proposing scalable extended technologies but faces many unsolvable challenges. The capacity expansion of the chain is mainly based on the improvement of the blockchain architecture itself, which improves the synthesis processing capacity of the whole network by directly increasing the block capacity and improving the block output speed, mainly including various performance improvement schemes based on directed acyclic graph or fragmentation. However, this kind of scheme is limited by the number of nodes and composition in the network, so the performance improvement is limited. In addition, some schemes adopt new consensus mechanisms, which lack security analysis and proof, increasing the risk of blockchain centralization and security attacks.

## 5. Conclusion

According to the existing problems among biological organizations, this paper constructs a network model of the overall architecture of the drug packaging image system and discusses the sharing process. Combined with the advantages of blockchain and the ROMA integration platform, the feasibility of the network model is analyzed. After analysis, it is found that the drug packaging image based on blockchain and the ROMA integration platform has many advantages. ROMA integrated platform not only cooperates with Shenzhen Biology, Xinghai, Wulian, and Tongji University but also provides technical support all over the world. By cleaning up the zombie information system, promoting the integration of similar systems, and connecting the original equipment and systems, the cost can be effectively saved. Innovation sharing and application service mode: the integrated platform of ROMA and blockchain enables open sharing of biological data. It helps with data support and decision making and helps with urban development and industrial innovation. While the drug packaging image based on the blockchain and Rome integrated platform has many advantages, it still faces challenges. For example, the relevant laws and regulations at the legal level, the system specifications at the management level, and the standards at the data level are not perfect; in the process of docking with the blockchain smart contract, its design and implementation are also facing difficulties, which requires a lot of attempts.

The article "Drug Packaging Management Based on the Effect of Medical Images on the Intracellular Polysaccharide Synthesis and Antivertigo Activity of Phalaenopsis" was published in 2021. Journal: J Healthc Eng.

## Figures and Tables

**Figure 1:** The compact DNA structure exhibited by bacteria.

**Figure 2:** P2P spread and the trend of ROMA.

**Figure 3:** The difference in sugar content of different polysaccharides.

**Figure 4:** The influence of chemical ions on the content of polysaccharides.

**Figure 5:** The content of intracellular polysaccharides in a single hormonal sac.

**Figure 6:** Multiomics data and bioinformatics analysis.

**Figure 7:** The relationship between *Phellinus esculentus* and high-concentration polysaccharides.

**Figure 8:** Phellinus xylinus encounters high concentrations of polysaccharides.

**Table 1:** Relative values of biosynthetic mechanisms.

Genome	Transcriptome	Proteome	Multiomics	epsN	Gene cluster	Key enzyme
Oxychloride	2.09	2.7	1.46	3.02	2.78	2.95
Algae cell	2.32	3.01	5.23	5.8	2.81	3.44
Carotene	2.67	1.41	1.64	5.64	2.07	2.82
Duncan	1.46	3.86	3.9	3.67	4.22	2.27
ANOVA	4.83	4.23	6.05	6.45	3.77	5.84
Strong acid	5.47	3.66	3.6	2.56	6.66	1.51

**Table 2:** Extracellular polysaccharide content of a single algal cell.

Genome	Oxychloride	Algae cell	Carotene	Duncan	ANOVA	Strong acid
Transcriptome	2.09	2.32	2.67	1.46	4.83	5.47
Proteome	2.7	3.01	1.41	3.86	4.23	3.66
Multiomics	1.46	5.23	1.64	3.9	6.05	3.6
Gene cluster	2.78	2.81	2.07	4.22	3.77	6.66
Key enzyme	2.95	3.44	2.82	2.27	5.84	1.51

## Data Availability

Data sharing is not applicable to this article as no datasets were generated or analyzed during the current study.
